The article "Development and Evaluation of a Simple and Effective Prediction Approach for Identifying Those at High Risk of Dyslipidemia in Rural Adult Residents" was retracted in 2021. Reasons: no approval from a third party; copyright claims.

# Development and Evaluation of a Simple and Effective Prediction Approach for Identifying Those at High Risk of Dyslipidemia in Rural Adult Residents

**DOI:** 10.1371/journal.pone.0043834

**Published:** 2012-08-28

**Authors:** Chong-Jian Wang, Yu-Qian Li, Ling Wang, Lin-Lin Li, Yi-Rui Guo, Ling-Yun Zhang, Mei-Xi Zhang, Rong-Hai Bie

**Affiliations:** 1 Department of Epidemiology and Biostatistics, College of Public Health, Zhengzhou University, Zhengzhou, Henan, People’s Republic of China; 2 Department of Clinical Pharmacology, School of Pharmaceutical Science, Zhengzhou University, Zhengzhou, Henan, People’s Republic of China; 3 Department of Endocrinology, Military Hospital of Henan Province, Zhengzhou, Henan, People’s Republic of China; Universidad Peruana Cayetano Heredia, Peru

## Abstract

**Background:**

Dyslipidemia is an extremely prevalent but preventable risk factor for cardiovascular disease. However, many dyslipidemia patients remain undetected in resource limited settings. The study was performed to develop and evaluate a simple and effective prediction approach without biochemical parameters to identify those at high risk of dyslipidemia in rural adult population.

**Methods:**

Demographic, dietary and lifestyle, and anthropometric data were collected by a cross-sectional survey from 8,914 participants living in rural areas aged 35–78 years. There were 6,686 participants randomly selected into a training group for constructing the artificial neural network (ANN) and logistic regression (LR) prediction models. The remaining 2,228 participants were assigned to a validation group for performance comparisons of ANN and LR models. The predictors of dyslipidemia risk were identified from the training group using multivariate logistic regression analysis. Predictive performance was evaluated by receiver operating characteristic (ROC) curve.

**Results:**

Some risk factors were significantly associated with dyslipidemia, including age, gender, educational level, smoking, high-fat diet, vegetable and fruit intake, family history, physical activity, and central obesity. For the ANN model, the sensitivity, specificity, positive and negative likelihood ratio, positive and negative predictive values were 90.41%, 76.66%, 3.87, 0.13, 76.33%, and 90.58%, respectively, while LR model were only 57.37%, 70.91%, 1.97, 0.60, 62.09%, and 66.73%, respectively. The area under the ROC cure (AUC) value of the ANN model was 0.86±0.01, showing more accurate overall performance than traditional LR model (AUC = 0.68±0.01, *P*<0.001).

**Conclusion:**

The ANN model is a simple and effective prediction approach to identify those at high risk of dyslipidemia, and it can be used to screen undiagnosed dyslipidemia patients in rural adult population. Further work is planned to confirm these results by incorporating multi-center and longer follow-up data.

The article "Development and Evaluation of a Simple and Effective Prediction Approach for Identifying Those at High Risk of Dyslipidemia in Rural Adult Residents" was retracted in 2021. Reasons: no approval from a third party; copyright claims.

## Introduction

Dyslipidemia is a widely recognized risk factor for cardiovascular diseases, a leading cause of death in both developed and developing countries [1], [2]. The World Health Organization (WHO) estimates that dyslipidemia is associated with more than half of the global cases of ischemic heart disease and more than four million deaths per year [3]. Evidence demonstrates that dyslipidemia can be prevented and controlled, which is cost-beneficial and with effective prevention programs can decrease the incidence and mortality of cardiovascular diseases [4], [5].

Estimating an individual’s risk across a range of presumed risk factors is fundamental to prevent dyslipidemia [6]. Due to its complex and multifactorial nature, the prevention of dyslipidemia must refer to multiple risk factors. Evidence showed that some predictors are associated with the occurrence of dyslipidemia [7]. Factors related to diet, lifestyle and family history might be associated with an increased risk of dyslipidemia [8], [9]. However, it is difficult to evaluate an individual’s risk of dyslipidemia when many predictors exist concomitantly. A model that integrates related factors and predicts the risk of dyslipidemia would be helpful to promote health education and counseling, and enable further development of computerized medical decision support systems for aiding healthcare practitioners to assess the risks of their patients quickly, inexpensively, and noninvasively [9], [10].

Logistic regression (LR) is often used to identify significant factors that correlate with disease, and has commonly been used to develop models for clinical diagnosis and treatment [11]. Artificial neural network (ANN) is a computer modeling technique based on the observed behaviors of biological neurons [12]. This is a non-parametric pattern recognition method that can recognize hidden patterns between independent and dependent variables [13]. Although ANN has been used in oncology, diabetes, hypertension, and other diseases [14]–[21], none have developed and evaluated the feasibility of the ANN model for predicting the risk of dyslipidemia in rural adults. Thus, it is unclear whether the ANN model is reliable and effective to identify those at high risk of dyslipidemia. Therefore, the purpose of this study was to develop and deliver an ANN model without biochemical parameters to identify those at high risk of dyslipidemia in rural adult population, and evaluate the predictive performance of the ANN model in comparison with the traditional LR model.

The article "Development and Evaluation of a Simple and Effective Prediction Approach for Identifying Those at High Risk of Dyslipidemia in Rural Adult Residents" was retracted in 2021. Reasons: no approval from a third party; copyright claims.

## Participants and Methods

### Study Population

This study was a cross-sectional survey, and subjects were selected randomly from eligible candidates in the residential registration record from the rural areas in Henan Province, China. The eligibility of the candidate was defined as those who were stable residents for at least 10 years in the study areas aged 35–78 years, and were free from the following conditions: 1) severe psychological disorders, physical disabilities, cancer, Alzheimer’s disease, or dementia, within 6 months; or 2) currently diagnosed with tuberculosis, acquired immune deficiency syndrome (AIDS), and other infectious diseases. Ultimately, a total of 8,914 residents who met the criteria enrolled in the study. Informed consent was obtained from all participants. The procedure of the study was approved by the Zhengzhou University Medical Ethics Committee, and written informed consent was obtained for all participants.

### Data Collection and Measurements

A home interview was conducted by physicians or public health workers from the local Centers for Disease Control and Prevention and the community hospital. All investigators and staff successfully completed a training program that oriented them both to the aims of the study and to the specific tools and methodologies used. At the training sessions, interviewers were given detailed instructions on administration of the study questionnaire.

#### Demographic data

Education level was classified into five categories: no education, primary school, middle school, high school, college and above. Marital status was categorized as unmarried, married/cohabitation, and divorced/widowed. Occupation was categorized as farmers, laborers, professionals and employers/managers. Individual annual income was calculated by total household income divided by the number of family members. Positive family history was defined as the participant’s parents or siblings having a history of dyslipidemia at or before the baseline examination.

#### Dietary and lifestyle behaviors

Three-day dietary intake data were collected from each subject using a 24-hour diet recall and a 2-day diet record. The daily intake of energy, nutrients, food and food groups for each subject were calculated using China Food Composition Table [22]. According to the Chinese Dietary Guidelines [23], vegetable and fruit intake was defined as consuming an average of more than 500 g per day, and fat intake is defined as consuming an average of more than 25 g per day.

Current smoking status included smoker and non-smoker. Participants who currently smoked and had smoked at least 100 cigarettes during their lifetime were classified as current smokers if they answered affirmatively to the following questions: “Do you smoke cigarettes now?” and “Have you smoked at least 100 cigarettes during your lifetime?” Physical activity level was classified as low, moderate, or high according to the International Physical Activity Questionnaire (IPAQ) scoring protocol [24].

The article "Development and Evaluation of a Simple and Effective Prediction Approach for Identifying Those at High Risk of Dyslipidemia in Rural Adult Residents" was retracted in 2021. Reasons: no approval from a third party; copyright claims.

#### Anthropometric data

Body weight and height were measured twice in light indoor clothing without shoes to the nearest 0.1 kg and 0.1 cm, respectively. Waist circumference (WC) was measured twice at the mid-point between the lowest rib and the iliac crest to the nearest 0.1 cm, after inhalation and exhalation. Central obesity based on WC (Male: WC ≥90 cm; Female: WC ≥80 cm) was defined according to WHO criteria for the Asia-Pacific region population [25].

#### Laboratory measurement

An overnight fasting blood specimen was collected in a vacuum tube containing EDTA for measurement of lipid profile. Blood specimens were centrifuged at 4°C and 3,000 rpm for 10 minutes, and the plasma was transferred and stored at −20°C for biochemical analyses. Total cholesterol (TC), triglycerides (TG), high-density lipoprotein cholesterol (HDL-C), and low-density lipoprotein cholesterol (LDL-C) were measured enzymatically on an automatic biochemical analyzer (Hitachi 7080, Toky, Japan) with reagents purchased from Wako Pure Chemical Industries (Osaka, Japan).

### Definition of Dyslipidemia

According to the China Adult Dyslipidemia Prevention Guide (2007 Edition) criteria [26], subjects were considered normal if their TC was less than 6.22 mmol/L, TG was less than 2.26 mmol/L, and HDL-C was greater than 1.04 mmol/L at the time of examination. The subjects were considered having dyslipidemia if one of their TC, TG or HDL-C were greater than 6.22 mmol/L, 2.26 mmol/L, or less than 1.04 mmol/L, respectively.

### Training and Validation Data Sets

Of 8,914 participants who met inclusion criteria, 75% of subjects (N1 = 6,686) were randomly selected to provide the training group for constructing ANN and LR prediction models. The remaining 25% of participants (N_2_ = 2,228) were assigned to the validation group for performance comparisons of ANN and LR models. The proportion of dyslipidemia between the training group and validation group was similar to the surveyed population data, and there was no statistically significant difference by χ^2^ test for gender and age between the training and validation datasets (Table 1).

**Table 1:** Comparison of baseline characteristics between the training and validation groups.

Variable	Participants (*N* = 8,914)		*P* value
	Training group (*N_1_* = 6,686)	Validation group (*N_2_* = 2,228)	
Age (years), mean (±sd)	53.89 (10.89)	52.56 (11.02)	0.9906
Gender (women), n (%)	3,712 (55.52)	1,276 (57.27)	0.1491
Occupation, n (%)			
Farmers	5,238 (78.34)	1,750(78.56)	0.9610
Laborers	586 (8.76)	191(8.57)	
Employers/managers	862 (12.89)	287(12.88)	
Education, n (%)			0.2317
No education	1,177 (17.60)	369 (16.56)	
Primary school	2,384 (35.66)	768 (34.47)	
Middle school	2,484 (37.15)	887 (39.81)	
High school	579 (8.66)	181 (8.12)	
College and above	62 (0.93)	23 (1.03)	
Marital status, n (%)			
Unmarried	34 (0.51)	9 (0.40)	0.8261
Married/cohabitation	6,126 (91.62)	2,043 (91.70)	
Divorced/widowed	526 (7.87)	176 (7.90)	
Physical activity, n (%)			
Low	1,913(28.61)	619(27.78)	0.4386
Moderate	1,579(23.62)	555(24.91)	
High	3,194(47.77)	1,054(47.31)	
Individual income (annual), mean (±sd)	2,075(1199)	2,037(1226)	0.1009
Waist circumference (cm), mean (±sd)	82.61(10.36)	82.46(10.15)	0.5222
TC (mmol/L), mean (±sd)	4.56 (0.96)	4.58 (0.95)	0.9492
TG (mmol/L), mean (±sd)	1.90 (0.53)	1.87 (0.65)	0.1052
H-DLC (mmol/L), mean (±sd)	1.11 (0.25)	1.17 (0.27)	0.1464
L-DLC (mmol/L), mean (±sd)	2.59 (0.79)	2.62 (0.77)	0.4164
Dyslipidemia, n (%)	3,115 (46.59)	1,011(45.38)	0.3200

The article "Development and Evaluation of a Simple and Effective Prediction Approach for Identifying Those at High Risk of Dyslipidemia in Rural Adult Residents" was retracted in 2021. Reasons: no approval from a third party; copyright claims.

### Modeling Tools

#### Logistic regression

The LR model generates the coefficients for the following formula used in logit transformation for predicting the probability of an event among patients with certain characteristics of interest: Logit (*P*) = *β_0_*+*β_1_ χ*_1_+*β_2_ χ_2_*+…+ *β_i_ χ_i_* [9]. The formula *P* = 1/(1+e^-logit(*P*)^) used for calculating the probability of dyslipidemia in this study, where 1 =  dyslipidemia and 0 =  non-dyslipidemia. A stepwise algorithm was used to construct the multivariate LR model. At each step, independent variables not yet included in the equation were tested for possible inclusion. The variable with the strongest significant contribution to improving the model was included. Variables already included in the logistic regression equation were tested for exclusion on the basis of a likelihood ratio test. The analysis ended when no further variables for inclusion or exclusion were available [27]. Furthermore, LR was used to estimate the coefficients (β) of these variables, from which the probability of dyslipidemia was estimated.

#### Artificial neural network

The ANN is a nonlinear statistical data modeling tool that can be used to model complex relationships between inputs and outputs or to find patterns in data. The processing elements or nodes are arranged in “input,” “hidden,” and “output” layers, each layer containing one or more nodes. The input layer consists of the data thought to be of value in predicting the outputs of the model [28], [29]. Each data point is represented by a node in the input layer. The output layer estimates the probability of the outcome as determined by the model. Each layer comprises one or more processing elements all interconnected in a way that each node in the hidden layer is connected to each node in the input and output layers [28], [29]. Each connection carries a “weight” or value that determines the relevance of a particular input for the resulting output [28], [29]. The ANN makes predictions based on the strength of connections between the neurons in the input, hidden, and output layers [28], [29]. The results of the output layer in ANN model represent the probability of a characteristic of interest (dyslipidemia). Figure 1 presents a flow chart describing the basic ANN design. A procedural description of the algorithm used for ANN in this study is available from the author and listed in Text S1. A more detailed description of ANN could be provided by Zou and Dumont [30], [31].

The article "Development and Evaluation of a Simple and Effective Prediction Approach for Identifying Those at High Risk of Dyslipidemia in Rural Adult Residents" was retracted in 2021. Reasons: no approval from a third party; copyright claims.

**Figure 1:** Framework of artificial neural network model for predicting an individual’s risk of dyslipidemia. The input layer contained 9 neurons. In the hidden layers, the numbers of neuron were 21. The output layer had only one neuron representing the probability of dyslipidemia. **Abbreviations:** X_A_, age; X_G_, gender; X_EL_, educational level; X_S_, smoking; X_HFD_, high-fat diet; X_VFI_, vegetable and fruit intake; X_FH_, family history of dyslipidemia; X_PA_, physical activity; X_WC_, waist circumference.

### Statistical Analysis

Analysis was performed in three stages. Firstly, a set of indicators contributing to the prediction of dyslipidemia was identified by univariate and multivariate logistic regression analysis based on the training group. Secondly, The ANN and LR models were performed with the probability of having dyslipidemia as the dependent variable and the risk factors as the independent variables. In general, the analysis structure of the neural network included three layers: input layer to accept information, hidden layer to process information, and output layer to calculate responses. In this study, the ANN model used the same input variables as the LR model. Thirdly, predictive performance was assessed by using receiver operating characteristic (ROC) curve analysis.

The LR model and ROC curve analysis were constructed using SAS 9.1 (SAS Institute, USA). The ANN model was performed with MATLAB 7.1 (MathWorks Institute, USA). All reported *P*-values were two-sided, and *P*-values less than 0.05 were considered statistically significant.

## Results

### Characteristics of the Participants

Table 1 shows the characteristics of the 8,914 subjects in the training and validation groups. The mean age (±sd) was 53.89±10.89 and 52.56±11.02 years in these two groups, respectively, while the number of females were 3,712 (55.52%) and 1,276 (57.27%), respectively. The prevalence rates of dyslipidemia were 46.59% and 45.38% in the training and validation groups, respectively. The relevant variables did not significantly differ between training and validation groups (*P*>0.05), confirming the reliability of random subject selection.

The article "Development and Evaluation of a Simple and Effective Prediction Approach for Identifying Those at High Risk of Dyslipidemia in Rural Adult Residents" was retracted in 2021. Reasons: no approval from a third party; copyright claims.

### Predictors of Dyslipidemia Risk

Table 2 shows the predictors of dyslipidemia risk identified from LR analysis based on the training group (*N_1_* = 6,686). With the construction of a multivariable model (LR analysis, the independent predictors were included when *P*<0.05, and were eliminated when *P*>0.1). Factors significantly associated with dyslipidemia were age (odds ratio *OR* = 1.042), higher-educational level (*OR* = 1.362), smoking (*OR* = 1.165), more high-fat diet (*OR* = 1.403), positive family history of dyslipidemia (*OR* = 1.876), and central obesity (Male: WC ≥90 cm; Female: WC ≥80 cm) (*OR* = 2.327). There was also an inverse relationship for male gender (*OR* = 0.758), more vegetable and fruit intake (*OR* = 0.844), and more physical activity (*OR* = 0.924).

**Table 2:** Multivariate logistic regression analysis on risk factors of dyslipidemia in the training group.

Variable	*β*	S.E.	*Wald*	*P*-value	*OR* (95%*CI*)
Age, X_A_	0.0410	0.0029	203.5210	0.0001	1.042 (1.036–1.048)
Male, X_G_	−0.2774	0.0800	12.0404	0.0005	0.758 (0.648–0.886)
Higher-educational level, X_EL_	0.3092	0.0609	25.7535	0.0001	1.362 (1.209–1.535)
Smoking, X_S_	0.1529	0.0454	11.3361	0.0008	1.165 (1.066–1.274)
More high-fat diet, X_HFD_	0.3385	0.1063	10.1416	0.0014	1.403 (1.139–1.728)
More vegetable and fruit intake, X_VFI_	−0.1701	0.0548	9.6278	0.0019	0.844 (0.758–0.939)
Positive family history, X_FH_	0.6290	0.0671	87.8728	0.0001	1.876 (1.645–2.139)
More physical activity, X_PA_	−0.0786	0.0321	5.9851	0.0144	0.924 (0.868–0.984)
Central obesity, X_wc_	0.8444	0.0561	226.3747	0.0001	2.327 (2.084–2.597)

**Abbreviations:** X_A_, age; X_G_, gender; X_EL_, educational level; X_S_, smoking; X_HFD_, high-fat diet; X_VFI_, vegetable and fruit intake; X_FH_, family history of dyslipidemia; X_PA_, physical activity; X_WC_, waist circumference.

### Prediction Models

The logit probability of having dyslipidemia was described by the following LR model: −2.7155+0.0410 X_A_ − 0.2774 X_G_ +0.092 X_EL_ +0.1529 X_S_ +0.3385 X_HFD_ - 0.1701 X_VFI_ +0.6290 X_FH_ - 0.0786 X_PA_ +0.8444 X_WC_. According to the predictors of dyslipidemia risk from the LR analysis, the ANN model was built using the training group data. The predictors used as the model input were X_A_, X_G_, X_EL_, X_S_, X_HFD_, X_VFI_, X_FH_, X_PA_, and X_WC_. The probability of whether an individual had dyslipidemia was the output variable. The analysis structure of the neural network included three layers: input, hidden and output layers. Figure 1 shows the input layer with 9 neurons, 21 hidden layer neurons and one output layer neuron, corresponding to the forecast variable (that is the probability of having dyslipidemia).

The article "Development and Evaluation of a Simple and Effective Prediction Approach for Identifying Those at High Risk of Dyslipidemia in Rural Adult Residents" was retracted in 2021. Reasons: no approval from a third party; copyright claims.

### Comparison of Predictive Performance

The ANN and LR models could successfully distinguish an individual’s risk of having dyslipidemia. We compared the individual’s predicted risk from the two models with the actual status using the validation group (*N_2_* = 2,228). The ANN model detected 911 dyslipidemia patients from the 1011 actual dyslipidemia patients, whereas the LR model only detected 582 dyslipidemia subjects. Figure 2 summarizes the ROC curve obtained from the LR and ANN models. For the ANN model, the sensitivity, specificity, positive likelihood ratio (+ LR), Negative likelihood ratio (− LR), positive predictive value (PPV), and negative predictive value (NPV) were 90.41%, 76.66%, 3.87, 0.13, 76.33%, and 90.58%, respectively, while the corresponding numbers were only 57.37%, 70.91%, 1.97, 0.60, 62.09%, and 66.73% in the LR model, respectively (Table 3). The AUC value of the ANN model was significantly higher (AUC = 0.86±0.01, 95% *CI*: 0.85–0.88) than that of the LR model (AUC = 0.68±0.01, 95% *CI*: 0.66–0.70) (*P*<0.001).

**Figure 2:** ROC curves of ANN and LR prediction models in the validation group. Areas under ROC curves were 0.86 and 0.68 for ANN and LR models, respectively. Area under ROC curve obtained by ANN was superior to that obtained by LR. **Abbreviation:** ANN, artificial neural network; LR, logistic regression; ROC, receiver operating characteristic.

## Discussion

To our knowledge, this is the first study to develop and evaluate the reliability and effectiveness of the ANN model for predicting dyslipidemia risk of rural adults in comparison with the LR model. Our findings showed that the ANN model had superior predictive performance, and the sensitivity, specificity, PPV, NPV, and AUC value of the ANN model were significantly higher than that of the traditional LR model. The ANN model can be used to identify undiagnosed dyslipidemia patients in rural adult population.

**Table 3:** Performance comparison of ANN and LR models for predicting dyslipidemia in the validation group.

Variable	ANN model	LR model	
Sensitivity (%, 95% *CI*)	90.41 (88.40–92.22)	57.37 (54,31–60.38)	
Specificity (%, 95% *CI*)	76.66 (74.18–79.03)	70.91 (68.29–73.50)	
+ LR (95% *CI*)	3.87 (3.42–4.40)	1.97 (1.71–2.28)	
− LR (95% *CI*)	0.13 (0.10–0.16)	0.60 (0.54–0.67)	
PPV (%, 95% *CI*)	76.33 (74.47–78.93)	62.09 (59.33–66.00)	
NPV (%, 95% *CI*)	90.58 (86.24–94.26)	66.73 (61.70–70.53)	
AUC (95% *CI*)	0.86 (0.85–0.88)	0.682 (0.66–0.70)	

***Abbreviation:*** *ANN, artificial neural network; LR, logistic regression; CI, confidence intervals; AUC, areas under ROC curve; + LR, positive likelihood ratio; − LR, Negative likelihood ratio; PPV, positive predictive value; NPV, negative predictive value.*

The article "Development and Evaluation of a Simple and Effective Prediction Approach for Identifying Those at High Risk of Dyslipidemia in Rural Adult Residents" was retracted in 2021. Reasons: no approval from a third party; copyright claims.

Because of the rapidly increasing prevalence of dyslipidemia, detecting people with undiagnosed dyslipidemia is very important in both public health and clinical practice [32], [33]. Lipid profile measurement is a standard method for identifying and diagnosing dyslipidemia [34], [35], but it is not available in resource limited settings, especially in some rural areas of developing countries. For example, the costs of TC, TG, HDL-C, and LDL-C measurement are more than ¥30 in China, which is probably the income of three days to a Chinese peasant. Therefore, an effective and inexpensive identifying approach has been sought which could be used to screen undiagnosed dyslipidemia in resource limited countries and areas. In this study, we used a general epidemiology survey database without biochemical parameters to develop and evaluate a prediction model to distinguish patients with dyslipidemia, which is not only inexpensive, but also quick and noninvasive.

Model sensitivity and specificity are important when testing whether a model can accurately recognize positive and negative outcomes [9]. The ideal model has both high sensitivity and high specificity [36]. In this study, the results of the predictive performance showed that the ANN model could be used to accurately screen undiagnosed dyslipidemia patients because it had sufficient sensitivity (90.41%) and specificity (76.66%) compared to the standard LR model (57.37% and 70.91%) for identifying true positive or negative patients. Since AUC provides a superior performance index in addition to superior accuracy, it was often used to evaluate the predictive accuracy of classifiers [37]. The AUC of a classifier can be defined as the probability of the classifier ranking a randomly chosen positive example higher than a randomly chosen negative example, and higher AUC values can be interpreted as higher predictive accuracy [37], [38]. For ANN model, the AUC value (AUC = 0.86±0.01) was superior to that of the LR model (AUC = 0.68±0.01) in terms of predictive accuracy. The above comparisons confirm that the sensitivity, specificity, and AUC for the prediction model constructed using ANN were significantly higher than that of the traditional LR model. That is, the ANN model outperforms the traditional LR model for predicting individual’s risk of dyslipidemia in rural adult residents.

The article "Development and Evaluation of a Simple and Effective Prediction Approach for Identifying Those at High Risk of Dyslipidemia in Rural Adult Residents" was retracted in 2021. Reasons: no approval from a third party; copyright claims.

The availability of the predictors is also very important when evaluating whether a model is feasible to identify positive and negative outcomes. This study examined the feasibility of the predictors of dyslipidemia in rural adult population. The findings based on the training dataset revealed nine common parameters significantly associated with dyslipidemia, including age, gender, educational level, smoking, high-fat diet, vegetable and fruit intake, family history, physical activity, and central obesity. These predictors without biochemical parameters were readily accessible in the rural population through routinely collected data in general practice or from general survey. In addition, the ANN predictive model can be easily navigated using a simple questionnaire through computerized medical decision support systems, in which the path depends on simple yes or no questions. The final result will help rural healthcare practitioners to quickly determine the individual’s risk of dyslipidemia. The ANN predictive model using demographic, lifestyle and anthropometric data provides a feasible approach to screen undiagnosed dyslipidemia patients in rural adult population.

Although this is the first study to develop and evaluate the feasibility of the ANN model for predicting individual’s risk of dyslipidemia in rural adult residents, study limitations should be noted. Firstly, evaluations of the different models were based on a cross-sectional survey without a longer follow-up period. Secondly, the samples were limited geographically and ethnically, consisting of a rural community of individuals aged 35–78 years old. Thirdly, the relevant variables were measured, such as smoking, physical activity, waist circumference, fat, vegetable and fruit consumption, on only a single occasion. Finally, the prediction model was based on a sample without use of data from multiple regions. Despite these limitations, the results are based on a large population-based study combining multiple risk factors, and the prediction approach was reliable and effective to screen undiagnosed dyslipidemia patients in rural adult residents.

### Conclusion

Our findings demonstrate that the ANN model had superior predictive performance compared with the traditional LR model to quickly identify those at high risk of dyslipidemia, and it can be used to screen undiagnosed dyslipidemia patients in rural adult population using general survey data or routinely collected data in general practice. This will help rural healthcare practitioners to evaluate the risks of their patients quickly, inexpensively, and noninvasively. Meanwhile, further work is planned to assess the utility of incorporating multiple rural locations and longer follow-up data.

The article "Development and Evaluation of a Simple and Effective Prediction Approach for Identifying Those at High Risk of Dyslipidemia in Rural Adult Residents" was retracted in 2021. Reasons: no approval from a third party; copyright claims.

## Supporting Information

Text S1 **This file contains the procedure of the artificial neural network model in the Matlab environment.**
(DOCX)
